The article "Effect of Routine Therapy Assisted by Physical Exercise on Pulmonary Function in Patients with Asthma in Stable Stage: A Systematic Review and Meta-analysis of Randomized Clinical Trials" was published in 2022. Journal: Comput Math Methods Med.

# Effect of Routine Therapy Assisted by Physical Exercise on Pulmonary Function in Patients with Asthma in Stable Stage: A Systematic Review and Meta-analysis of Randomized Clinical Trials

**DOI:** 10.1155/2022/2350297

**Published:** 2022-06-14

**Authors:** Xionghui Li, Chengye Mao, Yunchang Pan

**Affiliations:** Respiratory Department, The Sanming First Hospital Affiliated to Fujian Medical University, Sanming, Fujian 365000, China

## Abstract

**Objective:**

This study is aimed at investigating the efficacy of physical exercise-assisted routine therapy on the pulmonary function of patients with stable asthma to provide clinical evidence and data support to guide disease management.

**Methods:**

Randomized controlled clinical trials of drug therapy and/or physical exercise for patients with stable asthma were retrieved from the China National Knowledge Infrastructure (CNKI), Wanfang database, Embase, PubMed, and Web of Science database. The studies published between January 2000 and June 2021 that met the criteria were included, and corresponding data were extracted. The meta-analysis was performed using the statistical software Stata 16.0. Statistical pooled effect sizes and 95% confidence intervals were calculated using a random-effects or fixed-effects model, as funnel plots were made with Begg's rank correlation method to evaluate publication bias.

**Result:**

This meta-analysis included 14 randomized controlled studies. Physical exercise-assisted treatment (experiment group) or routine therapy was associated with significantly elevated levels of forced expiratory volume in 1 second (FEV1) and forced vital capacity (FVC) (*P* < 0.05). As for the peak expiratory flow (PEF) level (*P* < 0.05), its level was significantly increased with physical exercise-assisted therapy compared with the conventional approach (*P* > 0.05). Subgroup analysis indicated that the FVC level in the experimental group was higher than that in the control group (*P* < 0.05) regardless of the adoption of aerobic exercise/anaerobic exercise. In regard to the FEV1 and PEE levels, aerobic exercise was associated with elevated levels in the experimental group (*P* < 0.05), while no significant difference in anaerobic exercise between both groups was observed (*P* > 0.05). Further, FEV1, FVC, and PEF levels in the experimental group were higher than those receiving conventional treatment in the control group (*P* < 0.05).

**Conclusion:**

Routine treatment combined with physical exercise could improve the levels of FEV1, FVC, and PEF in patients with bronchial asthma in the nonacute attack stage and enhance pulmonary functions. As a safe and efficient adjuvant therapy, physical exercise can contribute to an improved prognosis and quality of life for patients with asthma.

## 1. Introduction

Asthma often manifests recurrent respiratory symptoms such as chest tightness, cough, shortness of breath, and wheezing, which are characterized by chronic airway inflammation, airway hyperreactivity, bronchoconstriction, and excessive mucus secretion, with great heterogeneity in its severity and duration [1]. Asthma is the most common chronic respiratory disease, with an incidence twice that of chronic obstructive pulmonary disease. Its global prevalence has increased by 13% from 1990 to 2015 and currently affects more than 358 million people worldwide [2]. In China, its overall prevalence among people aged 20 years and above reaches 4.2%, representing approximately 45.7 million people [3]. Severe asthma can be life-threatening and is responsible for about 300,000 deaths each year worldwide [4].

The etiology of asthma is multifactorial but mainly relates to genetic and environmental factors. Its pathological manifestations include chronic airway inflammation accompanied by infiltration of proinflammatory cells such as eosinophils, lymphocytes, and mast cells as well as shedding of airway epithelial cells [5, 6]. Long-term inflammation can impair the airways and induce airway remodeling, leading to basement membrane epithelial fibrosis, smooth muscle hypertrophy, and hyperplasia of the submucosal glands [7]. Therefore, asthma management and treatment are aimed at alleviating airway hyperresponsiveness and airflow limitation by eliminating airway inflammatory triggers, relieving inflammation with medical treatment, and widening narrow airways [8]. At present, inhaled corticosteroids (ICS) are the most effective drugs for asthma. They can be used in combination with long-acting beta-agonists (LABA) and long-acting muscarinic antagonists (LAMAs) in moderate to severe asthma patients [9–11]. Although asthma-related disability and mortality have decreased by approximately half in some developed countries such as the United States, Canada, the United Kingdom, France, Germany, and France between 2001 and 2015 due to the widespread use of ICS, their long-term use can lead to significant side effects. Asthma control is suboptimal in most patients with moderate to severe chronic asthma [12].

The Global Initiative for Asthma (GINA) guidelines propose that the goal of treatment is to attain complete or partial control of asthma, that is, to reduce the number of acute attacks of asthma, relieve clinical symptoms, and maintain patients in a stable phase through effective treatment measures [13]. Further, physical exercise also has the advantage that it can be flexibly performed at the patients' will as long as they are comfortable with the exercise intensity and can be easily accepted by adults or even the parents of children. Physical exercise has been reported to improve asthma symptoms, quality of life, exercise capacity, bronchial hyperresponsiveness, exercise-induced bronchoconstriction, and cardiorespiratory health and reduce nocturnal asthma symptoms, making asthma more manageable [14–16]. It has also been shown that aerobic training could improve aerobic capacity and significantly reduce the use of medications in patients with moderate to severe asthma [17]. In addition, aerobic training is beneficial in reducing eosinophil numbers and nitric oxide levels in the sputum of patients with moderate or severe persistent asthma, especially in patients with high levels of inflammation [18].

However, because asthma can also be induced by transient airway stenosis caused by a dramatic increase in the amount of air entering the respiratory tract during exercise, the effect of physical exercise on the improvement of lung function in asthma remains controversial [19–21]. The most common barrier to exercise in asthma is that it can trigger asthmatic symptoms. However, a study by Garfinkel et al. showed that asthma severity and methacholine challenge were not predictive of maximal oxygen uptake as a marker of aerobic fitness, suggesting that the severity of asthma should not be a cause to not perform physical activities [22]. Thus, we hypothesize that as long as an individualized dose of antiasthmatic drugs is combined with a healthy amount of exercise, a combination of the two could reduce the number of drugs needed or even the frequency of asthmatic exacerbations, thereby potentially decreasing the risks or severity of adverse events related to long-term pharmacological treatment.

This study is aimed at investigating the effects of drug therapy assisted by physical exercise on the pulmonary function of patients with stable asthma. Relevant randomized controlled trial studies were selected for this meta-analysis to evaluate the changes in pulmonary function before and after drug therapy and auxiliary physical exercise treatment.

## 2. Materials and Methods

### 2.1. General Information

This study collected and sorted relevant clinical trials published between January 2000 and June 2021, and their data were analyzed and summarized to comprehensively determine the effects of physical exercise-assisted routine treatment on the pulmonary functions in patients with stable asthma.

### 2.2. Method

#### 2.2.1. Literature Search Strategy and Database

In this paper, the search time was set from January 2000 to June 2021, and “asthma”, “exercise”, and “lung” were used as subject terms. Relevant clinical studies were screened from the Chinese National Knowledge Infrastructure (CNKI), Wanfang, Embase, PubMed, and Web of Science databases. There were no language and experimental design limitations during the search, and articles that met the study topics were included.

#### 2.2.2. Inclusion Criteria

(1) Study type: the study type is a clinical randomized controlled trial comparing the effects of routine drug therapy and drug therapy assisted by physical exercise on pulmonary function in patients with bronchial asthma. (2) Study subjects: all patients included were clinically diagnosed with bronchial asthma in the nonacute attack stage. (3) Intervention measures: patients were divided into a control group and an experimental group based on their health status and subjective wishes to appropriately increase physical exercise. The control group was given conventional drugs to treat chronic persistent bronchial asthma; on the basis of drug treatment in the control group, the experimental group was given increased physical exercise, including jogging, basketball, swimming, yoga, Tai Chi, cycling, physical training, and other aerobic or anaerobic exercises. (4) Outcome measures: the outcome measures were forced expiratory volume in the first second (FEV1), forced vital capacity (FVC), and peak expiratory flow (PEF).

#### 2.2.3. Exclusion Criteria

(1) The study design was inconsistent, and the diagnostic criteria or intervention measures were not clear; (2) the key data of the literature were missing, vague, and unable to be converted and combined, and relevant materials could not be obtained even after contacting the authors; (3) duplicated studies or the full text could not be obtained; (4) the literature was a systematic review, case report, conference paper, animal experiment, etc.

#### 2.2.4. Literature Screening and Data Extraction

First, all the retrieved literature was searched for duplicate checking manually and the EndNote software. Then, two researchers screened the literature according to the inclusion and exclusion criteria, read the original text, and extracted the relevant clinical data. In this process, if the researchers disagreed on a screened literature, a third researcher would decide and participate in the discussion and negotiation to obtain consistent final screening results. Finally, the researchers summarized the included literatures and extracted the relevant information such as literature title, author, publication year, type of study design, basic characteristics of study subjects, sample size, intervention measures, and outcome measures.

### 2.3. Statistical Analysis

In this study, the included data were analyzed using the Stata 16.0 software. The standard mean difference (SMD) and 95% confidence intervals (CI) were used to express continuous variables. The statistical heterogeneity among all studies was evaluated using the *χ*^2^ test. *P* < 0.05 and *I*^2^ ≥ 50% indicated significant heterogeneity among studies where the random-effects model was applied for meta-analysis. The fixed-effects model was used instead in the cases of homogeneity among studies with *P* > 0.05 and *I*^2^ < 50%, as subgroup analysis was conducted to analyze possible causes of heterogeneity. In this meta-analysis, the statistical results were presented by forest plots. When the number of final included studies was ≥10, Begg's method was used to draw the funnel plot for publication bias analysis. *P* < 0.05 indicated that the results were statistically significant.

## 3. Results

### 3.1. Literature Search Results

In this study, 1113 studies were obtained after a preliminary search in the indicated databases. Of them, 224 were excluded after removing duplicated publications. After screening and assessing eligibility, a total of 14 studies were found to meet the study inclusion criteria and were used for qualitative analysis [18, 23–35]. The detailed screening process and results are shown in Figure 1. The studies' characteristics are shown in Table 1.

### 3.2. Meta-analysis Results of the Effects of Physical Exercise on Pulmonary Function in Patients with Asthma

#### 3.2.1. Forced Expiratory Volume in 1 Second (FEV1)

All clinical studies included in this meta-analysis utilized FEV1 to assess the effects of routine treatment assisted by physical exercise on pulmonary function in patients with asthma. Of these, 13 studies examined FEV1 levels before and after treatment in the experimental and control groups [18, 23–26, 28–35], while 1 only reported on FEV1 levels in asthmatic patients after treatment [27]. In the experimental group, the meta-analysis of FEV1 levels before and after the treatment incorporating physical exercise showed significant heterogeneity among the studies (*I*^2^ = 91.6%, *P* < 0.001), so the random-effects model was adopted for analysis. The result suggested that incorporating auxiliary physical exercise into the treatment was associated with a significantly elevated FEV1 level, as shown in Figure 2(a). Similarly, the meta-analysis of FEV1 levels before and after routine treatment in the control group also demonstrated notable heterogeneity among the studies (*I*^2^ = 88.1%, *P* < 0.001). The random-effects model suggested that routine treatment also increased the FEV1 levels of asthma patients, which was significantly different between the two groups (SMD = −0.69, 95% CI (-1.09, -0.30), *P* = 0.001) (Figure 2(b)).

The present study divided the different types of physical activity in the experimental group into the aerobic and anaerobic exercise groups to perform a subgroup analysis of FEV1 levels in both groups. The 13 [18, 23–26, 28–35] studies compared the experimental group with the control group before treatment, and as their overall results showed homogeneity among the studies (*I*^2^ = 0.0%, *P* = 0.855), the fixed-effects model analysis was used. Before treatment, the FEV1 level gap between the two groups was not significantly different among the studies (SMD = 0.07, 95% CI (-0.05, -0.20), *P* = 0.251). To compare FEV1 levels after treatment between the two groups in 14 [18, 23–35] studies, the experimental group of 6 [23–26, 33, 35] studies used anaerobic exercise. Our meta-analysis indicated no significant heterogeneity among the studies when comparing FEV1 levels after anaerobic exercise and conventional treatment (*I*^2^ = 0.0%, *P* = 0.652). As a consequence, the fixed-effects model analysis was utilized for analysis. The results indicated no statistical difference in the FEV1 level between anaerobic exercise and routine treatment (SMD = 0.12, 95% CI (-0.10, 0.33), *P* = 0.281). Analysis of another 8 [18, 27–32, 34] studies in which the experimental group adopted aerobic exercise indicated significant heterogeneity among various studies in terms of the FEV1 level after treatment (*I*^2^ = 71.4%, *P* = 0.001). As shown by the random-effects model, aerobic was associated with a relatively high FEV1 level (SMD = 0.41, 95% CI (0.11, 0.71), *P* = 0.008). We then comprehensively evaluate the efficacy of aerobic and anaerobic exercise with routine treatment. The overall results of this meta-analysis on FEV1 levels after treatment in the two groups indicated significant heterogeneity among the studies (*I*^2^ = 62.8%, *P* = 0.001). The random-effects model was used and demonstrated that physical exercise was associated with significantly higher FEV1 levels than the routine asthma treatment (SMD = 0.29, 95% CI (0.08, 0.51), *P* = 0.007) (Figure 2(c)).

#### 3.2.2. Forced Vital Capacity (FVC)

A total of 13 [18, 23–26, 28–35] studies reported on the FVC levels of the experimental and control group before and after treatment to further assess the efficacy of routine treatment and physical exercise on pulmonary functions in asthma. Significant heterogeneity among the studies was observed by meta-analysis of FVC levels in the experimental group before and after treatment (*I*^2^ = 91.5%, *P* < 0.001). The random-effects model has then revealed that combination with physical exercise significantly elevated FVC levels (SMD = −0.77, 95% CI (-1.23, -0.31), *P* = 0.001) (Figure 3(a)). In the control group of the included studies, FVC levels before and after routine treatment also indicated significant heterogeneity (*I*^2^ = 87.8%, *P* < 0.001). The random-effects model showed that the FVC level of asthma patients was significantly improved with routine treatment (SMD = −0.52, 95% CI (-0.91, -0.13), *P* = 0.009) (Figure 3(b)).

Next, we analyzed the impact of aerobic and anaerobic exercise. Subgroup analysis of the FVC levels of asthma patients before and after treatment was performed. We found that 13 [18, 23–26, 28–35] studies compared the experimental group with the control group before treatment, and the overall results indicated significant heterogeneity among the studies (*I*^2^ = 64.3%, *P* = 0.001) with no significant difference in the FVC level before treatment (SMD = 0.19, 95% CI (-0.03, 0.41), *P* = 0.090). All 14 [18, 23–35] studies measured FVC levels of asthma patients receiving different treatments, including 6 studies analyzing the effect of anaerobic exercise. We noticed a significant heterogeneity in the FVC levels after anaerobic exercise or routine treatment among the studies (*I*^2^ = 57.0%, *P* = 0.040). The results of random-effects model analysis demonstrated that anaerobic exercise was associated with higher FVC levels in patients (SMD = 0.34, 95% CI (0.04, 0.68), *P* = 0.047). The other 8 [18, 27–32, 34] studies using aerobic exercise in the experimental group also showed significant heterogeneity between the two groups (*I*^2^ = 80.6%, *P* < 0.001). Random-effects model analysis showed that compared with routine treatment alone, combination of aerobic exercise and routine treatment had better improvement in FVC levels (SMD = 0.44, 95% CI (0.07, 0.81), *P* = 0.019). Further, comprehensive comparisons of FVC levels after treatment between the two groups displayed significant heterogeneity among the studies (*I*^2^ = 73.6%, *P* < 0.001). The model analysis showed that physical exercise could induce higher FVC levels than routine treatment (SMD = 0.41, 95% CI (0.15, 0.66), *P* = 0.002) (Figure 3(c)).

#### 3.2.3. Peak Expiratory Flow (PEF)

In 9 [18, 23, 25, 28, 30, 31, 33–35] studies, the PEF levels were measured in asthmatic patients upon different treatments. As shown in Figure 4(a), the meta-analysis indicated significant heterogeneity in the PEF levels before and after treatment in the experimental group (*I*^2^ = 86.9%, *P* < 0.001). The results of the random-effects model analysis revealed that the adoption of physical exercise based on routine treatment was associated with a higher level of PEF (SMD = −0.60, 95% CI (-1.03, -0.18), *P* = 0.006).  Figure 4(b) illustrates the PEF levels before and after conventional treatment in the control group, and our meta-analysis showed significant heterogeneity among the studies (*I*^2^ = 86.5%, *P* < 0.001). The random-effects model showed no significant difference in PEF levels after conventional treatment (SMD = −0.13, 95% CI (-0.56, -0.30), *P* = 0.557).

Next, we analyzed the impact of aerobic and anaerobic exercise on asthma based on PEF levels. The PEF level of asthma patients before treatment was detected first. The overall results suggested significant heterogeneity between different studies (*I*^2^ = 91.0%, *P* < 0.001). The random-effects model showed no significant difference in PEF levels between the two groups before treatment among the studies (SMD = 0.47, 95% CI (-0.07, 1.01), *P* = 0.091). Of 10 [18, 23, 25, 27, 28, 30, 31, 33, 34] studies that compared PEF levels after two different treatments, 4 [23, 25, 33, 35] took anaerobic exercise apart from routine treatment in the experimental group. Meta-analysis comparing PEF levels in both groups showed significant heterogeneity among the studies (*I*^2^ = 61.9%, *P* = 0.049). The difference in PEF levels between two groups did not reach significance (SMD = 0.18, 95% CI (-0.24, 0.60), *P* = 0.395). In the other 6 [18, 27, 28, 30, 31, 34] studies, aerobic exercise was used in the experimental group. Our analysis showed significant heterogeneity in the PEF level after treatments among different studies (*I*^2^ = 95.3%, *P* < 0.001), and the presence of aerobic exercise was largely associated with the PEF level (SMD = 1.27, 95% CI (0.30, 2.24), *P* = 0.010). Then, the PEF level after treatment was comprehensively compared between the two groups. The overall meta-analysis results revealed heterogeneity among the studies (*I*^2^ = 92.4%, *P* < 0.001). The random-effects model combined analysis suggested that the PEF level of asthma patients in the experimental group was significantly higher (SMD = 0.69, 95% CI (0.11, 1.28), *P* = 0.020) (Figure 4(c)).

### 3.3. Analysis of Publication Bias

Publication bias analysis was performed for FEV1 and FVC levels of the experimental and control groups before and after treatment and for the experimental group versus the control group after treatment (Figures 5 and 6). Begg's rank correlation test indicated no significant publication bias in the meta-analysis (*P* > 0.05). The asymmetric distribution of scatter points on both sides of the funnel plot indicated that the study sample distribution was uneven, suggesting the possibility of publication bias in the included studies. The inclusion of some studies with small sample size, low-quality literature, and other factors could have led to the observed potential publication bias results.

## 4. Discussion

Long-term use of ICS, LABA, and LAMAs has been associated with side effects, while physical exercise was shown to strengthen respiratory muscles, improve bronchiolar patency, reduce airway inflammation, and thus could effectively improve pulmonary function [36, 37]. As a result, exercise therapy and drug therapy are included as one of the recommended asthma therapies in the GINA guidelines [38]. The physical exercise modality and training intensity are key factors for improving lung function [13, 39], but the clinical application of aerobic and anaerobic exercise with different intensities remains controversial. Most studies suggest that clinical trials for chronic respiratory diseases should focus on regular aerobic training programs of moderate-intensity rather than high-intensity anaerobic exercise, as it can trigger exercise-induced asthma [40, 41]. Further, the official research consensus of the American Thoracic Society and the European Respiratory Society also recommends 30 minutes of moderate-intensity physical exercise for pulmonary rehabilitation [42].

Vital capacity plays a crucial role in diagnosing and assessing disease severity in asthma and is closely related to cardiopulmonary function [43, 44]. Few earlier exercise training studies have considered lung function as the primary outcome measure and thus were insufficient to assess the effectiveness of asthma interventions. FEV1, FVC, and PEF are the three most common indicators for objective evaluation of pulmonary function in patients with asthma, of which FVC has been shown to greatly hinge on respiratory muscle function, lung compliance, and airway resistance as well as the overall health status of patients. The GINA guidelines propose spirometry for the management of asthma exacerbations requiring emergency treatment or hospitalization. The reference values for FEV1 and PEF are taken as a reflection of admission and treatment [45], as they also reflect airway patency and are used to measure airway function and respiratory muscle strength, thereby indicating the degree of airway obstruction and lesion [43, 46]. This study demonstrated that physical exercise therapy could significantly improve FEV1, FVC, and PEF levels in patients with asthma. In a study by Eichenberger et al. [47], the authors reported that exercise therapy only increased FEV1 levels rather than PEF levels. This difference might be related to pooling between newly published studies and differences in interventions between different studies. This meta-analysis showed that routine treatment assisted by physical exercise could increase FEV1, FVC, and PEF levels and effectively improve the pulmonary function of patients with asthma, which has a positive guiding effect for clinical nondrug treatment of asthma.

The limitations of this study were the limited number of eligible studies, the presence of heterogeneity and publication bias, and the inclusion of both Chinese or English literature which could have some possibility of language bias, since different detection methods were used for the outcome measures. Thus, to provide more concrete evidence on the efficacy of exercise in the treatment of stable asthma, higher-quality clinical studies with larger cohorts of patients should be performed in a more standardized manner.

## 5. Conclusions

Collectively, physical exercise combined with routine treatment had a significantly positive effect on stable asthma patients, as the combination treatment could improve the patients' FEV1, FVC, and PEF levels, thereby improving their pulmonary function. For the prevention and management of asthma, physical exercise could be a safe and efficient adjuvant therapy to improve the patients' treatment efficacies and quality of life on the basis of conventional treatment. Further, it should be clarified that physicians should recommend appropriate physical exercise for asthma patients, which could help maintain physical health, improve asthma symptoms, and enhance their quality of life.

## Figures and Tables

**Figure 1:** A flow chart of literature search of this study.

**Figure 2:** Forest plot analysis of FEV1 in the two groups: (a) forest plot of FEV1 level before and after treatment in the experimental group; (b) forest plot of FEV1 level before and after treatment in the control group; (c) forest plot of FEV1 level after treatment in the experimental group compared with the control group.

**Figure 3:** Forest plot analysis of FVC in the two groups: (a, b) forest plot of FVC level before and after treatment in the experimental group (a) and the control group (b); (c) forest plot of subgroup analysis of FVC level after aerobic and anaerobic exercise in the experimental group and conventional treatment of asthma in the control group. FVC: forced vital capacity.

**Figure 4:** Forest plot analysis of PEF in the two groups: (a, b) forest plot of PEF level before and after treatment in the experimental group (a) and control group; (c) forest plot of subgroup analysis of the PEF level after aerobic and anaerobic exercise in the experimental group and control group. PEF: peak expiratory flow.

**Figure 5:** Funnel plot analysis of FEV1 in the two groups: (a, b) funnel plot of FEV1 level before and after treatment in the experimental group (a) and the control group (b); (c) funnel plot of comparison of FEV1 level of patients after treatment in the experimental and control group.

**Figure 6:** Funnel plot of FVC level in the two groups: (a–c) funnel plot of FVC level before and after treatment in the experimental group (a) and the control group (b) and contract of FVC level in the experimental group after treatment with the control group (c).

**Table 1:** Basic characteristics of included literature.

Study	Year of publication	Sample time (year.month)	Cases Exp/Con	Age (years)		Sex (male/female)		Movement measures	Treatment time (weeks)	Study design	Outcome measures
				Exp group	Con group	Exp group	Con group				
Yang et al. [35]	2020	2017.8-2019.10	53/52	8.2 ± 1.3	8.7 ± 1.4	34/19	32/20	Bicycle kick	8	RCT	①②③
Li et al. [33]	2016	2015.2-2015.6	22/22	11.9 ± 2.3	12.5 ± 3.0	NR	NR	Bicycle kick	8	RCT	①②③
Basaran et al. [28]	2006	NR	31/31	10.4 ± 2.2	10.5 ± 2.1	20/11	20/11	Basketball	8	RCT	①②③
Liao et al. [27]	2019	2014.1-2014.10	25/15	8.3 ± 0.3	8.0 ± 0.3	14/11	7/8	Taijiquan activity	12	RCT	①②③
Mendes et al. [18]	2011	NR	27/24	25.7-47.3	22.0-47.5	3/24	6/18	Yoga	12	RCT	①②③
Wang and Hung [26]	2009	NR	15/15	9-11	9-11	10/5	10/5	Swimming	6	RCT	①②③
van Veldhoven et al. [25]	2001	NR	23/24	10.5 ± 1.2	10.7 ± 1.2	16/7	18/6	Gym strength training	12	RCT	①②③
Xu [32]	2021	2017.6-2020.2	25/25	43.1 ± 13.7	41.1 ± 12.2	12/13	14/11	Setting up exercise	12	RCT	①②③
Li and Shii [34]	2021	2018.1-2018.10	39/39	50.9 ± 4.8	51.0 ± 5.1	21/18	23/16	Setting up exercise	12	RCT	①②③
Li et al. [30]	2015	2013.8-2014.8	64/64	8.8 ± 2.4	8.8 ± 2.4	35/29	34/30	Rope skipping, jogging	24	RCT	①②③
Wu [29]	2016	2015.1-2015.12	64/64	65.8 ± 2.8	65.2 ± 2.9	34/30	34/30	Setting up exercise	24	RCT	①②③
Gao [31]	2020	2018.6-2019.6	60/60	40.6 ± 11.4	40.9 ± 11.8	31/29	29/31	Setting up exercise	NR	RCT	①②③
Wicher et al. [24]	2010	2004.11-2009.8	30/31	10.4 ± 3.1	10.9 ± 2.6	12/18	15/16	Swimming	12	RCT	①②③
Arandelović et al. [23]	2007	NR	45/20	33.1 ± 9.8	33.6 ± 10.9	34/11	15/5	Swimming	24	RCT	①②③

Note: Exp: experimental; Con: control; RCT: randomized controlled trial; NR: not reported; ①: forced expiratory volume in one second (FEV1); ②: forced vital capacity (FVC); ③: peak expiratory flow (PEF).

## Data Availability

The datasets used and analyzed in this study are accessible upon request from the corresponding author.

## Abbreviations

CNKI: China National Knowledge Infrastructure
FEV1: Forced expiratory volume in 1 second
FVC: Forced vital capacity
PEF: Peak expiratory flow
ICS: Inhaled corticosteroids
LABA: Acting beta-agonists
LAMAs: Long-acting muscarinic antagonists
GINA: Global Initiative for Asthma
SMD: Standard mean difference
CI: Confidence intervals.
